# Analysis of Strategies and Skills of English Translation Based on Coverage Mechanism

**DOI:** 10.1155/2022/7767045

**Published:** 2022-07-21

**Authors:** Bin Liu, Jing Wang

**Affiliations:** ^1^School of Foreign Studies, Suqian University, Jiangsu, Suqian 223800, China; ^2^College of Education, Taylor University, Subang Jaya 47500, Selangor, Malaysia

## Abstract

In order to alleviate the problem of over translation and missing translation in NMT, based on the consistency and complementarity of information stored in different covering models, a multicoverage fusion model is proposed, which uses coverage vector and coverage score to guide the attention mechanism at the same time. First, the concept level definitions of words are covered. Then, two kinds of translation history information stored in the cover vector and cover score are used to guide the calculation of the attention score at the same time. Finally, the dual attention decoding method based on the fusion coverage mechanism is adopted. The experimental results show that the multicoverage fusion model can improve the translation quality of NMT.

## 1. Introduction

Due to the diversity and complexity of natural languages, it is still difficult to translate one language properly into another. At present, neural machine translation (NMT) has shown great potential under the condition of large corpus and computational capacity and has developed into a new machine translation method [1, 2]. This method requires only bilingual parallel corpus, which is convenient for training large-scale translation models. It not only has high research value but also has a strong industrialization ability, which has become a hot spot in current machine translation research [3].

Neural machine translation based on encoder and decoder structure is a general model, which is not fully designed for the machine translation task itself, so there are still some problems to be solved. It requires bilingual dictionaries to be fixed in size. Considering the complexity of training, dictionary size, and sentence length are usually limited to a small range [4, 5]. As a result, NMT is faced with more severe problems of unknown words and long sentences. Only bilingual training data are used, and no additional prior knowledge is required, such as large-scale monolingual corpus, annotated corpus, and bilingual dictionary. In addition, the structural characteristics of machine translation make it difficult to use external resources. Monolingual corpus, annotated corpus, bilingual dictionary, and other resources can significantly improve translation quality in statistical machine translation [6], but prior knowledge has not been fully applied overtranslation and inadequate translation are the problems of NMT. The overlay mechanism is a common method in statistical machine translation to ensure the integrity of the translation. It is difficult to directly model the covering mechanism in NMT [7]. The attention mechanism is a significant improvement on NMT, but its deficiency is that historical attention information is not taken into account in the generation of target language words, and the constraint mechanism is weak. In addition, in some cases, the generation of target language words does not need to pay too much attention to the source language information. For example, in Chinese-English translation, when the function word “The” is generated, more attention should be paid to the target language information. In addition, there are problems of OverTranslation and UnderTranslation in NMT [8], and the existing attention mechanism also needs to be improved. Although the above-given methods can alleviate the problems of over translation and missing translation in NMT to a certain extent, due to the structural characteristics of a word for word prediction of the NMT model cannot be completely avoided.

Therefore, in this paper, firstly, the problems of existing coverage models and the possibility of fusion between different methods are analyzed. Then, multiple coverage information fusion methods are used to record translation history information complementary to guide the calculation of attention weight, which can reduce the loss of historical information updating and improve the distribution of attention weight, so as to inhibition the phenomenon of over translation and missing translation.

## 2. Translation Model Based on Fusion of Multiple Coverage Strategies

### 2.1. Basic Ideas

The covering idea is proposed in the phrase based statistical machine translation model. In each decoding, all untranslated phrases and their translation results are added to the candidate set. Whenever a phrase translation result is added to the output sequence, the corresponding source language phrase should be marked as “translated,” which ensures that each source language phrase is covered by translation, and is not translated repeatedly.

Covering information is also very important for NMT. Due to the lack of a covering mechanism in the NMT model, it is an effective method to improve the over translation and missing translation problem by adding a covering mechanism to the NMT model.

Specifically, assuming that a sentence sequence of the source language *X*={*x*_1_, *x*_2_, *x*_3_, *x*_4_, *x*_5_} is given, Its initial coverage set *C*={0,0,0,0,0}. Among them, “0” indicates that the corresponding source language word has not been translated, while “1” indicates that the source language word has been covered by translation. In addition, assuming that the corresponding target phrase source language phrase {*x*_2_, *x*_3_, *x*_4_} is {*y*_*m*_,…, *y*_*n*_}, then after {*y*_*m*_,…, *y*_*n*_} is added to the translation output sequence, the overlay set will be updated to *C*={0,1,1,1,0}. If it is specified that a phrase can only be translated once in the process of translation, then follow this step to translate until the translation is completed, and the overlay set should be *C*={1,1,1,1,1}. At this point, the phrase and the source language are effectively translated only once.

### 2.2. Coverage Model

#### 2.2.1. Covering Vector

In the statistical machine translation model, all source language phrases can only be translated once, so its coverage mechanism is a hard alignment. However, the attention mechanism of the NMT model is a kind of soft alignment; that is, the words covered by attention are still allowed to participate in the prediction of the next word. Therefore, it is very difficult to model the coverage mechanism directly [9]. In Literature [6], a covering model is proposed, in which a covering vector is set up to explicitly store the historical coverage information of each word in the source language sentence. In order to provide historical information for the translation process, the coverage vector is incorporated into the original attention mechanism model, where more attention is allocated to untranslated words and the weight of translated words is reduced. The structure of the coverage vector guided attention model is shown in Figure 1.

After fusing the covering vector, the calculation method of the attention mechanism is as follows:

(1) $$\begin{array}{c} e_{i,j}=a\left(t_{j-1},h_{i},{\text{CV}}_{i,j-1}\right)\\ =v_{a}^{T}\tan h\left(W_{a}t_{j-1}+U_{a}h_{i}+V_{a}{\text{CV}}_{i,j-1}\right). \end{array}$$

Among them, *CV*_*i*,*j*−1_ represents the coverage vector corresponding to the source language word *x*_*i*_ before time *j*, and *V*_*a*_ is the weight matrix.

Since the history information changes after each step of decoding, the coverage vector of each source word needs to be updated. Its method is shown in the following equation:

(2) $$\begin{array}{c} {\text{CV}}_{i,j}=f\left({\text{CV}}_{i,j-1},a_{ij},h_{i},t_{j-1}\right), \end{array}$$

where *F*(·) is a recurrent neural network whose basic neural unit can use only a simple tanh layer or GRU with a more complex structure to capture long-distance dependencies.

#### 2.2.2. Coverage Score

It is used to indicate the degree of source language translation. If the translation results have high coverage of the source language words, the corresponding coverage score is also high; on the other hand, if the translation results have low coverage of the source language, the corresponding coverage score is also low. Suppose a sentence pair (*X*, *Y*) is given, the number of Chinese words in *X* and *Y* is expressed as |*X*| and |*Y*| separately. For any source language word *x*_*i*_, its coverage is defined as all target words *y*_*j*_ The sum of the attention scores of the words in the source language is shown in the following equation:

(3) $$\begin{array}{c} {\text{coverage}}_{x_{i}}=\sum_{j=1}^{\left|Y\right|}a_{ij}. \end{array}$$

On this basis, the coverage score of source language sentences is calculated by using the coverage of all source language words. The calculation method is shown in the following equation:

(4) $$\begin{array}{c} cs\left(X,Y\right)=\sum_{i=1}^{\left|X\right|}\log\;\varphi \left(\;{\text{coverage }}_{x_{i}},\beta \right). \end{array}$$

Among them, *β* is an adjustable parameter, *φ*(*·*) is truncation function. The coverage score is linearly combined with the original conditional probability function of the model to obtain the final evaluation function. The improved evaluation function is shown in the following equation:

(5) $$\begin{array}{c} \text{score}\left(X,Y\right)=a\cdot \;\log P\left(Y|X\right)+b\cdot \text{cs}\left(X,Y\right). \end{array}$$

Among them, log*P*(*Y|X*) represents the value of conditional probability predicted by the model, *a* and *b* represent an adjustable parameter used to balance the effect of conditional probability and coverage score. The introduction of the coverage score makes the model consider the coverage of source language sentences and reduce the bias of translation results of a short sentence.

### 2.3. Translation Model Based on Multiple Coverage Strategies

#### 2.3.1. Problem Description

Although the NMT model based on covering vector can alleviate the phenomenon of over translation and missing translation, this problem still exists. As shown in Figure 2, “Lavender” in the original text has been translated twice, while “Provence” has been omitted. When the first lavender is generated, the Coverage vector based NMT model mistakenly allocates more attention to lavender than Provence, which results in repeated translation and missing translation.

From the above-given examples, it can be seen that the NMT model based on covering vector still has further improvement space in attention allocation. As mentioned above, both coverage vector and coverage score can record the coverage information in the translation process in an explicit way. In the decoding stage, the former stores and updates the information abstractly in the form of a vector, calculate and guide the translation of attention through history; the latter is accumulated in the form of constant and used as the coverage of translation results for the selection of translation results. Compared with the coverage score, the coverage vector cannot directly quantify the coverage of translation results, and there is information loss when using GRU update; while it is difficult to determine the upper and lower limits of the coverage of each source language vocabulary with a fixed value, so it is impossible to compare the coverage between words.

#### 2.3.2. Model Decoding

Coverage vector and coverage score are complementary in the storage of coverage information. In order to combine the advantages of the two methods, this paper proposes a multicoverage fusion model which combines the coverage vector and the coverage score. The coverage score is used to reduce the impact of information loss when the coverage vector is updated, and improve the distribution of attention weight. The concept of word level coverage score is defined first. Then, according to the different fusion methods of coverage vector and coverage score, two kinds of multicoverage fusion models, hierarchical and parallel, are proposed. The overall framework is shown in Figure 3.

The coverage vector and the updated attention vector of each target word in the predicted sentence are obtained through the coverage mechanism layer. The coverage mechanism is shown in Figure 4.

During decoding, the attention weight vector *α*_*t*_^src^ of text is obtained from the hidden state *s*_*t*−1_ at the previous moment, the hidden state sequence H of the source language through the double attention mechanism layer. The key point of the coverage mechanism layer is to maintain a coverage vector *C*_*t*_ in the prediction project. It is the accumulative sum of attention distribution of all previous prediction steps, which records the historical information that the model has paid attention to and avoids focusing on repetitive information, as shown in the following equation:

(6) $$\begin{array}{c} C_{t}^{\text{src}}=\sum_{\hat{t}=0}^{t-1}\alpha_{t}^{\text{src}}. \end{array}$$

The obtained coverage vector is applied to the attention layer to obtain the updated attention weight, as shown in equations (7) and (8).

(7) $$\begin{array}{c} e_{t,i}^{\text{src}}={\left(v_{a}^{\text{src}}\right)}^{T}\tan h\left(U_{a}^{\text{src}}s_{t}+W_{a}^{\text{src}}h_{i}+V_{a}^{\text{src}}C_{t,i}^{\text{src}}\right). \end{array}$$

(8) $$\begin{array}{c} \alpha_{t,i}^{\text{src}}=\frac{\text{exp}\left(e_{t,i}^{\text{src}}\right)}{\sum_{j=1}^{N}\text{exp}\left(e_{t,j}^{\text{scc}}\right)}. \end{array}$$

Among them, tanh is the nonlinear activation function, *v*_*a*_^src^, *U*_*a*_^src^, *W*_*a*_^src^ are the parameters used for learning in the model. The weight *e*_*t*,*i*_^src^ can be interpreted as the correlation between the target word generated by the decoder and the source sequence word *x*_*i*_ at *t*. *α*_*t*,*i*_^scc^ represents the normalization of the obtained similarity score.

The coverage vector is added as an additional input to affect the prediction of the target language. Then, get the updated context attention vector *c*_*t*_. The text attention vector *c*_*t*_ at time *t* is obtained by the weighted sum of the source language implicit state sequence *h*_*i*_ and the weight *α*_*t*,*i*_^src^ obtained by the text attention model, as shown in the following equation:

(9) $$\begin{array}{c} c_{t}=\sum_{i=1}^{N}\alpha_{t,i}^{\text{src}}h_{i}. \end{array}$$

With the updated *i*_*t*_ as the additional input, the candidate implicit state *s*_*t*_′ is used, and the source language attention vector *c*_*t*_ calculates the final implicit state *s*_*t*_ at time *t*, as shown in equations (10)–(13).

(10) $$\begin{array}{c} z_{t}=\sigma \left(W_{z}^{src\;}c_{t}+U_{z}s_{j}^{\prime }\right), \end{array}$$

(11) $$\begin{array}{c} r_{t}=\sigma \left(W_{r}^{src\;}c_{t}+U_{r}s_{j}^{\prime }\right), \end{array}$$

(12) $$\begin{array}{c} {\underline{s}}_{t}=\tan h\left(W^{srr\;}c_{t}+r_{t}⊙\left(Us_{t}^{\prime }\right)\right), \end{array}$$

(13) $$\begin{array}{c} s_{t}=\left(1-z_{t}\right)⊙{\underline{s}}_{t}+z_{t}⊙s_{t}^{\prime }, \end{array}$$

where *z*_*t*_ is the renewal gate, *r*_*t*_ is the reset gate, ${\underline{s}}_{t}$ is the candidate hidden state, *s*_*t*_ is the final hidden state, *W*_*z*_^*src* ^, *U*_*z*_, *W*_*r*_^*src* ^, *U*_*r*_, *W*^*src* ^, *U* is the parameter used for learning in the model.

Finally, output the model, the prediction of the target word *y*_*t*_ at the *t* moment is related to the implicit state *s*_*t*_ of the target word at the current moment, the target word *y*_*t*−1_ generated by the prediction at the previous moment, and the text attention vector *c*_*t*_, as shown in the following equation:

(14) $$\begin{array}{c} P\left(y_{t}|y_{<t},C,A\right)=\text{softmax}\left(f\left(s_{t},y_{t-1},c_{t},i_{t}\right)\right)\propto ,\\ \text{exp}\left(L_{o}\text{tan}h\left(L_{s}s_{t}+L_{w}E_{y}\left[y_{t-1}\right]+L_{⊙}c_{t}+L_{c}i_{t}\right)\right), \end{array}$$

where *f* and softmax are nonlinear activation functions, and *L*_*o*_, *L*_*s*_, *L*_*w*_, *L*_*c*_, *L*_*ci*_ are parameters used by the model for learning.

## 3. Experiment and Analysis

### 3.1. Evaluation Method

BLEU (Bilingual Evaluation Understudy) algorithm evaluates translation performance by calculating the n-element words co-occurring in the translation result and the translation [10]. Firstly, MaxRefCount (n-gram) is calculated as the maximum number of possible occurrences of an n-word in a sentence. Then, it is compared with the number of occurrences of this n-word in the candidate translation, Count(n-gram), and the minimum value between them is taken as the final number of matches of this n-word. As shown in the following equation:

(15) $$\begin{array}{c} {\text{Count}}_{\text{clip}}\left(n-\text{gram}\right)=\text{min}\left\{\text{Count}\left(n-\text{gram}\right),\text{MaxRefCount}\left(n-\text{gram}\right)\right\}. \end{array}$$

And, then the precision *P*_*n*_ of the later co-occurrence n-element words is defined as follows:

(16) $$\begin{array}{c} P_{n}=\frac{\sum_{c\in \text{ candidates }}\sum_{n-\text{ gram }\in C}{\text{Count}}_{\text{clip }}\left(n-\text{gram}\right)}{\sum_{C\in \text{ candidates }}\sum_{n-\text{ grameC }}\text{Count}\left(n-\text{gram}\right)}. \end{array}$$

Since n-gram's matching degree tends to choose shorter sentences, a translation result that only translates part of the original sentence accurately will still have a high matching degree, BLEU introduces Brevity Penalty into the final scoring result to avoid the bias of scoring, as shown in the following equation:

(17) $$\begin{array}{c} \text{BP}=\left\{\begin{array}{c} 1,\;\text{ if }l_{c}>l_{s},\\ e^{1-l_{s}},\;\text{if }l_{c}\leq l_{s}, \end{array}\right. \end{array}$$

where *l*_*c*_ represents the length of the translation result, and *l*_*s*_ represents the length of the reference translation. When there are multiple references, the length closest to the translation result is selected as the length of the reference. It can be found that only when the length of the interpretation result is not exactly the length of the reference text will the punishment factor be presented.

BLEU usually only considers the accuracy of 4-GRAM at most, since the accuracy of n-gram statistics decreases exponentially with the increase of order. In order to balance the effect of statistics of each order, a geometric average is used for weighted summation, and then the length penalty factor is multiplied to obtain the final calculation formula as shown in the following equation:

(18) $$\begin{array}{c} \text{BLEU}=\text{BP}\times \text{exp}\left(\sum_{n=1}^{N}W_{n}\text{log}P_{n}\right), \end{array}$$

where *N* is the maximum order of n-element words, *W*_*n*_ is the weight coefficient, *N* = 4, *W*_*n*_ = 1/N.

### 3.2. Parameter Setting

About 6.5 million sentence pairs were extracted from the bilingual parallel corpus provided by CWMT2018. Using newsdev2017 as a validation set for parameter tuning and model selection that a total of 2002 sentences are included. Three datasets, newstest2017, cwmt2018, and newstest2018, were selected as test sets to verify the model, each containing 2000, 2481, and 3981 sentences. Before training and testing, the corpus is generalized, the word segmentation of the Chinese and English corpus is carried out by using the open-source tool of Niutrans, and the subword segmentation is carried out by using byte pair encoding.

The baseline system uses seq2seq, and the settings of the model are displayed in Table 1. The initial learning rate is set to 0.0001. In decoding, the beam search algorithm is adopted, and the length penalty, beam size, and length penalty coefficient are introduced and set to 15 and 1.3, respectively. 350000 steps were trained iteratively on the training set, and the 15 checkpoints with the highest BLEU are saved in the verification set for model testing. The coverage model based on the coverage vector is set up as the control. The coverage vector dimension is set to 10 and the GRU gate function is used to update. In the hierarchical multicoverage model, the balance coefficient is set to 0.5.

### 3.3. Result Analysis

During training, the 15 models with the highest BLEU were saved on the verification set corpus. In the test, the parameters are averaged first, and the final translation is generated on this basis. The specific experimental results are shown in Figure 5.

According to the experimental results in Figure 5, the average BLEU value of the baseline system on three test sets is 26.78%. On the basis of the baseline system, the coverage model has little improvement, and BLEU is only increased by 0.15%. The results of the two multicoverage fusion models are significantly improved compared with the baseline system and are better than the coverage model. The average BLEU of the HMC model was 27.43%. Compared with the baseline system and coverage model, BLEU increased by 0.65% and 0.5%, respectively; while the average BLEU value of the PMC model is 27.21%, which is 0.43% and 0.28% higher than the baseline system and coverage model, respectively. Compared with the two multicoverage models, the overall promotion effect of the HMC model is more obvious.

The interpretation impact of long sentences is one of the significant records to assess the exhibition of the NMT model. In order to research on the performance of the multicoverage fusion model in different source language sentence length intervals, the source dialects in the test set were assembled by the strategy for Reference [6], and the BLEU of the HMC model was compared with the baseline system and coverage model in the range of translation results on source language length (0, 10], (10, 20], (20, 30], (30, 40], (40, 50] and (50, +∞). The results are shown in Figure 6.

The performance of the HMC model is better than the baseline system and coverage model. Compared with baseline system, BLEU increased by 0.47%, 0.65%, 0.48%, and 0.79%, respectively, and on the basis of coverage model, it increased 0.22%, 0.55%, 0.44%, and 0.63%, respectively. Through the analysis of the corpus, it can be found that this length interval contains many fragments of long sentences after segmentation. The structure and meaning of these sentences are not complete enough, so the translation performance of the model is affected to a certain extent.

As shown in Figure 7, there are over translation problems in the Baseline system, Coverage model and HMC model, but the number of words in the translation of the coverage model and HMC model is less than that of the baseline system. Among them, the coverage model is 13.5% less than the baseline system, and the HMC model is further reduced by 10.5% on the basis of the coverage model, which shows that the HMC model can further alleviate the over translation problem in NMT on the basis of covering model.

In Figure 2, because the source language word “普罗旺斯Provence” wrongly establishes a corresponding relationship with “薰衣草Lavender,” which makes the word “薰衣草Lavender” appears in repeated translation. This problem is corrected in the HMC model, as shown in Figure 8. HMC model correctly translates “普罗旺斯薰衣草” into “Provence Lavender.”

## 4. Conclusion

Introducing coverage mechanism into the NMT model can alleviate the over translation and missing translation problems. However, the coverage information stored by the covering vector or coverage score is not perfect. Therefore, this paper discusses the information storage, usage, advantages, and disadvantages of different coverage models, and based on the consistency of translation history information and the complementarity between models, a multicoverage fusion model is proposed. Firstly, the concept of word level covering score is defined; Then, the information stored in the coverage score and coverage vector is used to guide the calculation of attention weight. According to the different fusion methods of coverage vector and coverage score, two methods, hierarchical multicoverage model and parallel multicoverage model, are proposed. The experimental results show that compared with the PMC model, the overall promotion effect of the HMC model is more obvious, and the multicoverage fusion method can further reduce the phenomenon of over translation and omission translation.

## Figures and Tables

**Figure 1:** Structure of coverage-based attention model.

**Figure 2:** An example of NMT model translation based on covering vector.

**Figure 3:** NMT model based on multicoverage.

**Figure 4:** Coverage mechanism.

**Figure 5:** BLEU of translation.

**Figure 6:** BLEU under different source language length.

**Figure 7:** Evaluation of repeated translation.

**Figure 8:** Solution of over translation problem.

**Table 1:** Parameters setting.

Parameter	Value
Neural network cell unit	LSTMCell
Encoder layers	2
Decoder layers	4
Dimension vector words	512
Hidden layer state dimension	512
Vocab	32 k
Batch_size	32
Max_length	50

## Data Availability

The dataset can be accessed from the corresponding author upon request.
